# Effects of Hydroxychloroquine on Proteinuria in IgA Nephropathy: A Systematic Review and Meta-Analysis

**DOI:** 10.1155/2021/9171715

**Published:** 2021-12-03

**Authors:** Jialing Zhang, Xiangxue Lu, Jianan Feng, Han Li, Shixiang Wang

**Affiliations:** Department of Blood Purification, Beijing Chao-Yang Hospital, Capital Medical University, Beijing 100020, China

## Abstract

**Introduction:**

The present meta-analysis was to explore the efficacy of hydroxychloroquine (HCQ) in IgA nephropathy patients in terms of proteinuria.

**Method:**

We systematically searched PubMed and Embase for studies that compared HCQ and other treatments to reduce proteinuria in patients with IgA nephropathy up to June 2021. Mean ± SD of percentage change and level of proteinuria was calculated.

**Results:**

A total of 5 studies with 587 participants were included. IgA nephropathy patients who received HCQ were at a lower level of mean proteinuria at 6 months. However, there was no statistical difference between HCQ and control group considering percentage reduction in proteinuria. The long-term therapeutic effect of HCQ might be inferior to HCQ and renin-angiotensin-aldosterone system inhibition.

**Conclusion:**

HCQ might play a role in the reduction of proteinuria in IgA nephropathy patients. The addition of HCQ to other immunosuppressive agents should be clarified further.

## 1. Introduction

IgA nephropathy, also known as Berger disease, is the most common primary glomerulonephritis and prevalent chronic glomerular disease in the world. About 40% of renal biopsies in Asia, 10% in the United States, and 20% in Europe show IgA nephropathy [1]. Immunofluorescence microscopy shows the deposition of IgA in the glomerular basement membrane, causing subsequent hematuria and progressive kidney disease. Proteinuria has been recognized as a risk factor for kidney function decline in kidney disease [2] and poor prognosis in IgA nephropathy [3].

The management of IgA nephropathy involved monitoring of blood pressure, proteinuria, hematuria, and estimated glomerular filtration rate (GFR). Renin-angiotensin-aldosterone system inhibition (RAASi) or angiotensin receptor blocker is recommended to slow proteinuria and lower blood pressure. Immunosuppression and corticosteroid can also benefit for heavy proteinuria. It was suggested that patients with persistent proteinuria ≥ 1 g/d and GFR > 50 mL/min per 1.73 m^2^ should receive a 6-month course of corticosteroid therapy [4]. However, corticosteroids should not be used for more than six months due to serious adverse effects [5, 6].

Hydroxychloroquine (HCQ), regarded as an immunomodulatory and anti-inflammatory agent, is a current therapeutic option for several autoimmune and rheumatic diseases, such as systemic lupus erythematosus and rheumatoid arthritis. Evidence suggests that HCQ can prevent organ damage [7] and thrombosis [8]. However, the definite effect of HCQ on proteinuria in IgA nephropathy patients was still on debate [9, 10]. Therefore, we conducted this meta-analysis to evaluate the efficacy of HCQ for proteinuria in IgA nephropathy patients.

## 2. Method

### 2.1. Search Strategy

This meta-analysis followed meta-analyses (PRISMA) guidelines [11]. The published study protocol is available at the PROSPERO registry (http://www.crd.york.ac.uk/PROSPERO/, CRD42021251836). Articles were identified via PubMed and Embase databases through June 2021. Studies suggesting treatment of HCQ for proteinuria in IgA nephropathy patients satisfied the inclusion criteria. Search terms for PubMed included ((((Hydroxychloroquine) OR (plaquenil)) OR (hydroxychlorochin)) AND (((((IgA nephropathy) OR (IgA glomerulonephritides)) OR (Berger's disease)) OR (Immunoglobulin A nephropathy)) OR (IgA type nephritis))) AND (((albuminuria) OR (proteinuria)) OR (microalbuminuria)) (search string for Embase available in Figure 1).

### 2.2. Selection Criteria

We included articles in English that met the eligibility criteria based on the PICOS strategy: (1) patients diagnosed with IgA nephropathy and being given HCQ, (2) compared HCQ with placebo or other immunosuppressive agents, (3) relevant outcomes included proteinuria level from baseline to the end of study, and (5) published randomized controlled trials and observational studies. Two reviewers independently screened for studies, and any disagreement in the literature screening or data extraction was resolved by a third reviewer through discussion. Reviewers also screened the reference list of review articles and other systematic reviews for other potentially relevant citations. A flowchart depicting the search strategy is presented in Figure 2.

### 2.3. Statistical Analysis

All statistical analyses were performed by Review Manager 5.3. Results presented in median (interquartile range) were transformed into mean ± SD according to formula [12, 13]. Statistical heterogeneity of the included studies was assessed using the *I*^2^ statistics [14]. Random-effect model was used to minimize the heterogeneity and external variance while *I*^2^ > 50%; otherwise, a fixed-effect model was employed. To further identify potential differences across the studies, subgroup analyses were conducted. The quality of studies was appraised using the Newcastle–Ottawa Scale (NOS) for assessing quality of nonrandomized trials in meta-analysis. Scores of 0 to 9 were allocated to each study. Scores of 6 and above were deemed to be of high quality. Sensitivity analyses were performed by removing each study stepwise, while publication bias was evaluated by funnel plot. A *p* < 0.05 represents statistical significance.

## 3. Results

### 3.1. Characteristics of the Studies Included in This Meta-Analysis

After a comprehensive search, 13 potentially relevant articles were totally screened in PubMed and Embase. Eight studies were removed because of duplication, nonrelevant, or desired outcomes. Finally, a total of 5 studies [9, 10, 15-17] were included in our meta-analysis aiming to evaluate the effect of HCQ on proteinuria in IgA nephropathy (placebo or other agents were used as control) (shown in Figure 2). Characteristics of participants and studies were described in Table 1. The mean age of participants ranged from 28.8 ± 10.2 to 42.2 ± 13.1 years, and the percentage of men varied across studies (range, 34.6-67%). Range of baseline proteinuria level from studies included in the meta-analysis was from 1.5 (1.2, 1.9) to 2.35 (1.54, 2.98) g/d. Three retrospective studies scored 6/9 on the NOS, and a remainder scored 7/9.

### 3.2. Clinical Outcomes

IgA nephropathy patients who received HCQ did not show a significant percentage reduction in proteinuria compared with those in the control group (shown in Figure 3). Although a random-effect model was employed, significant heterogeneity was identified across studies (*I*^2^ = 87, *p* < 0.00001). Sensitivity analysis indicated that results remained unchanged with the exclusion of any individual study (shown in Figure 4(a)). Another four studies [9, 10, 15, 16] performed that patients treated with a 6-month regimen for HCQ were at a lower mean proteinuria level compared with patients in the control group (SMD = −0.33, 95%CI = −0.50 to -0.16, *p* = 0.0002) (shown in Figure 5). No significant heterogeneity was identified across studies. Further sensitivity analysis indicated that the effect of HCQ on mean proteinuria level did not substantially differ with exclusion of any individual study (shown in Figure 4(b)). Publication bias was shown in funnel plot (shown in Figure 6).

### 3.3. Subgroup Analysis

Of the five studies, four studies [9, 10, 15, 16] compared the percentage reduction in proteinuria at 2, 4, and 6 months in the HCQ group to the control group, while one study [17] showed percentage reduction in proteinuria at 12 and 24 months. We performed a subgroup analysis according to the duration of treatment of HCQ, and significant differences were not observed in percentage reduction in proteinuria between HCQ and controls for 2, 4, and 6 months. However, we found IgA nephropathy patients treated with HCQ for more than 6 months were at a significantly lower percentage reduction in proteinuria (SMD = 27.42, 95%CI = 11.01 to 43.83, *p* = 0.001) (shown in Figure 7). Furthermore, considering three studies comparing the efficacy of HCQ and RAASi to RAASi only, two studies comparing HCQ to corticosteroid or conventional immunosuppressive agent, we also performed subgroup analysis according to the individual agent. Overall, nonsignificant difference was found (shown in Figure 8).

## 4. Discussion

In the current study, we compared HCQ with controls in IgA nephropathy patients in terms of the percentage change in proteinuria and mean proteinuria level. By meta-analysis of 5 studies, we found HCQ might play a slight role in reducing proteinuria in IgA nephropathy patients. However, the long-term effect of HCQ on percentage change in proteinuria was relatively poor.

IgA nephropathy is the most common primary glomerulonephritis worldwide [18]. IgA nephropathy can present with gross hematuria, nephrotic syndrome, chronic kidney disease, and rapidly progressive glomerulonephritis. IgA, mainly produced at mucosal surfaces, is mainly responsible for mucosal defense. Kidney biopsy remains the only way to diagnose IgA nephropathy with light microscopy, electron microscopy, and immunofluorescence. The main pathogenesis of IgA nephropathy is excess deposits of galactose-deficient IgA1 in serum and glomerular basement membrane, triggering circulating immune complexes accumulated in the mesangial cells, leading to mesangial proliferation, extracellular matrix synthesis, and podocyte damage. Considering high incidence of end-stage renal disease and mortality in IgA nephropathy patients, it is urgent to find an appropriate treatment plan in the clinical practice.

Measurement of proteinuria, an important factor for poor prognosis, offers a noninvasive method to risk stratify IgA nephropathy patients. A retrospective observational study reported kidney function of patients with time − averaged proteinuria > 1.0 g/day deteriorated faster than those with time − averaged proteinuria < 1.0 g/day [19]. Le et al. also confirmed that IgA nephropathy patients with time − averaged proteinuria > 1.0 g/day were associated with a 9.4-fold risk for renal failure than patients with time − averaged proteinuria < 1.0 g/day [20]. As a result, proteinuria might be an indicator to evaluate the efficacy of HCQ in patients with IgA nephropathy.

Previous meta-analysis has proved the combination of RAASi and steroid to reduce proteinuria effectively in IgA nephropathy patients [21, 22]. However, the investigation of HCQ was limited. Liu et al. [9] included 30 IgA nephropathy patients and found percentage change in proteinuria from baseline to 2, 4, and 6 months was significantly higher in the HCQ and RAASi group than that in the RAASi and placebo group. Yang et al. [16] also confirmed the efficacy of HCQ and RAASi on proteinuria reduction when compared to RAASi alone. In the current study, we found the mean proteinuria level at 6 months was significantly lower in the HCQ group than patients in the control group. Furthermore, the treatment of HCQ was relatively well tolerated by most patients with IgA nephropathy. No serious adverse events were documented during treatment with HCQ in the including articles. The mechanism of HCQ to reduce proteinuria in patients with IgA nephropathy was not clarified yet. HCQ is usually absorbed in the upper intestinal tract and eliminated in renal. It is widely accepted to accumulate in the lysosomes, probably due to its flat aromatic core structure and basic side chain. Accumulated HCQ might increase the local pH and inhibit the function of lysosomes which might involve in antigen processing and MHC class II presentation [23]. On the other hand, HCQ might block Toll-like receptor (TLR) signaling by directly binding to nucleic acids [24], which played a crucial role in the innate immune system. Furthermore, HCQ might also inhibit cytokine production by inhibiting TLR pathways. Willis et al. [25] have reported that HCQ resulted in a significant decrease in interferon-*α* level. Hjorton et al. [26] also showed that HCQ might interfere with cytokine production and gene expression in plasmacytoid dendritic cells and peripheral blood mononuclear cells. The effect of HCQ on B cell differentiation and T cell activation was also confirmed [27, 28].

In this meta-analysis, we included studies exploring the level of proteinuria in IgA nephropathy patients received HCQ. However, the difference of percentage reduction in proteinuria between HCQ and control group was not significant. We further performed a subgroup analysis according to the duration of HCQ, and no significant difference in the percent change in proteinuria was noted between two groups after received HCQ for 2, 4, and 6 months. The follow-up period was probably not long enough to draw a clear conclusion. In this meta-analysis, three studies compared HCQ and RAASi to RAASi only, while two studies compared HCQ to corticosteroid or conventional immunosuppressive agent. We found the efficacy of antiproteinuria was comparable between HCQ and other agents according to the subgroup analysis. Otherwise, we found the antiproteinuric effect of HCQ and RAASi was slightly inferior to that of RAASi alone for a >12-month regimen. A previous study also reported a slight benefit of corticosteroids compared to HCQ [10]. Meanwhile, in patients with proteinuria above 1 g/day, the antiproteinuric effect of HCQ and immunosuppressive agent was not significantly different from immunosuppressive treatment alone. Patients in the control group might have received other antiproteinuria agent before the study, which might overestimate the efficacy of treatment in the control group. Considering the sample size was relatively small, the results might not be stable enough. As a result, the effect of reducing proteinuria might be attenuated by duration of therapy, and the definite interaction of HCQ and other immunosuppressants on proteinuria should be explored by more large-scale randomized clinical trials in the future.

To our knowledge, this is the first meta-analysis to definite the efficacy of HCQ to reduce proteinuria in IgA nephropathy patients compared to other agents. In this meta-analysis, we performed subgroup analysis according to the duration of treatment and different agents in the control group. Although the superiority of HCQ to other agents was slight, we found the efficacy of HCQ might be modified by duration of treatment. Our study also has potential limitations. First, the number of studies included was relatively small. Although no serious adverse events were recorded in this study, more randomized clinical trials are preferred to clarify the efficacy and safety of HCQ. Second, studies in this meta-analysis only included IgA nephropathy patients from China. Despite of the high heterogeneity, we could not perform a subgroup analysis according to the race. Third, the effect of pathological types and renal function on treatment was not considered.

In conclusion, HCQ has a slight antiproteinuric effect in IgA nephropathy patients. The long-term effect of HCQ in addition to other immunosuppressants should be explicated further.

## Figures and Tables

**Figure 1:** Search strategy for Embase.

**Figure 2:** Flow diagram of the trail selection.

**Figure 3:** Forest plot of percentage reduction of proteinuria comparing HCQ and control.

**Figure 4:** Forest plot of sensitivity analysis ((a) sensitivity analysis for percentage reduction of proteinuria comparing HCQ and control; (b) sensitivity analysis for mean level of proteinuria at 6 months comparing HCQ and control).

**Figure 5:** Forest plot of mean level of proteinuria at 6 months comparing HCQ and control.

**Figure 6:** Funnel plot to assess the risk of publication bias.

**Figure 7:** Forest plot of subgroup analysis according to the duration.

**Figure 8:** Forest plot of subgroup analysis according to the type of agent.

**Table 1:** Baseline of characteristics of studies.

Author	Country	Study	HCQ group	Control group	Age (E/C) (year)	Male (E/C) (%)	Baseline proteinuria level (E/C) (g/d)	Percentage reduction in proteinuria	Median proteinuria level at 6 months (g/d)	NOS
Yang et al. 2019 [10]	China	Retrospective case-control	HCQ (0.2 g twice daily for eGFR > 45 ml/min/1.73 m^2^; 0.1 g twice or thrice daily for eGFR 30-45 ml/min/1.73 m^2^; 0.1 g once daily for eGFR 15-30 ml/min/1.73 m^2^) *N* = 92	Corticosteroid *N* = 92	37.0 ± 10.0 vs. 37.2 ± 12.6	50% vs. 50%	1.7 (1.2, 2.3) vs. 1.8 (1.3, 2.5)	2 months −28.0% (−50.8, −6.4) vs. -29.8% (−56.8, 12.9) 4 months −42.6% (−60.6, −25.0) vs. -42.3% (−72.1, −20.4) 6 months −48.5% (−62.6, −31.4) vs. -62.9% (−81.1, −34.9)	0.8 (0.6, 1.1) vs. 0.7 (0.3, 1.1)	6

Tang et al. 2020 [15]	China	Retrospective case-control	HCQ+IS (HCQ: 0.2 g twice daily for eGFR > 60 ml/min/1.73 m^2^; 0.1 g twice or thrice daily for eGFR 30-60 ml/min/1.73 m^2^; 0.1 g once daily for eGFR 15-30 ml/min/1.73 m^2^) *N* = 26	Conventional IS *N* = 26	28.8 ± 10.2 vs. 30.8 ± 12.2	34.6% vs. 38.5%	2.35 (1.47, 2.98) vs. 2.35 (1.54, 2.98)	2 months −40.17% (−48.71, −20.88) vs. −13.4% (−61.66,42.97) 4 months −33.62% (−49.15, −13.95) vs. −30.43% (−64.4, 0.00) 6 months −39.81% (−66.26, −12.37) vs. −31.99% (−67.08, −9.14)	1.10 (0.85, 1.61) vs. 1.24 (0.87, 2.58)	6

Liu et al. 2019 [9]	China	Randomized clinical trail	HCQ+RAASi (HCQ: 0.2 g twice daily for eGFR > 60 ml/min/1.73 m^2^; 0.1 g thrice daily for eGFR 45-60 ml/min/1.73 m^2^; 0.1 g twice daily for eGFR 30-45 ml/min/1.73 m^2^) *N* = 30	Placebo+RAASi *N* = 30	37.6 ± 11.6 vs. 35.6 ± 9.6	63% vs. 67%	1.6 (1.1, 2.2) vs. 1.9 (1.3, 2.6)	2 months −28.4% (−46.4, −11.4) vs. −1.4% (−29.2, 31.9) 4 months −38.0% (−58.4, −26.5) vs. −3.5% (−30.6, 29.2) 6 months −48.4% (−64.2, −30.5) vs. 10.0% (−38.7, 30.6)	0.9 (0.6, 1.0) vs. 1.9 (0.9, 2.6)	
Yang et al. 2018 [16]	China	Retrospective case-control	HCQ+RAASi *N* = 90	RAASi *N* = 90	37.3 ± 8.9 vs. 37.7 ± 10.8	48.9% vs. 47.8%	1.5 (1.2, 2.1) vs. 1.5 (1.2, 1.9)	6 months –43% (–57, –12) vs. –19% (–46, 17)	0.8 (0.7, 1.2) vs. 1.2 (0.8, 1.8)	6

Tang et al. 2021 [17]	China	Retrospective	HCQ+RAASi (HCQ: 0.2 g twice daily for eGFR > 60 ml/min/1.73 m^2^; 0.1 g thrice daily for eGFR 45-60 ml/min/1.73 m^2^; 0.1 g twice daily for eGFR 30-45 ml/min/1.73 m^2^; 0.1 g once daily for eGFR < 30 ml/min/1.73 m^2^) *N* = 77	RAASi *N* = 34	38.2 ± 10.1 vs. 42.2 ± 13.1	49.4% vs. 35.3%	1.55 (1.16, 2.23) vs. 1.56 (0.98, 2.37)	12 months −38.24% (−54.45, −14.26) vs. −52.05% (−81.87, −27.86) 24 months −35.69% (−70.33, −2.36) vs. −74.12% (−82.51, −58.30)		7

HCQ: hydroxychloroquine; eGFR: estimated glomerular filtration rate; E/C: experimental group/control group; RAASi: renin-angiotensin-aldosterone system inhibition; IS: immunosuppressive agent.
